The article "Elevated CEA and CA 19-9 Levels within the Normal Ranges Increase the Likelihood of CRC Recurrence in the Chinese Han Population" was retracted in 2023. Reasons: signs of a paper mill; suspected computer-generated content; unreliable results or conclusions; lack of ethics approval or compliance.

# Elevated CEA and CA 19-9 Levels within the Normal Ranges Increase the Likelihood of CRC Recurrence in the Chinese Han Population

**DOI:** 10.1155/2022/8666724

**Published:** 2022-09-22

**Authors:** Lujia Wang, Guangkai Zhang, Jiafeng Shen, Yujiang Shen, Guojun Cai

**Affiliations:** Department of Anus and Intestine, Hangzhou Ninth People's Hospital, Hangzhou, Zhejiang 310030, China

## Abstract

**Objective:**

This study aimed to determine if variations in the expression profiles of CA 19-9 and carcinoembryonic antigen (CEA) within the reference range could serve as possible biomarkers for postoperative CRC recurrence.

**Method:**

This retrospective cohort investigation enrolled 2,596 cases of CRC that received curative surgery. Serum CEA/CA 19-9 were measured through chemiluminescence immunoassay (CLIA).

**Results:**

During follow-up (median follow-up = 5.2 years), in total, 837 patients experienced recurrence. The fully adjusted hazard ratios (HRs) were significantly higher, ≥1 standard deviation (±SD), in patients with upregulated CEA/CA 19-9 levels (HRCEA = 7.06; HRCA 19 − 9 = 3.98) than in those with downregulated CEA/CA 19-9 levels. The likelihood of recurrence remained consistently greater in cases of elevated CEA/CA 19-9 levels during sensitivity analyses.

**Conclusions:**

The findings of this analysis showed that variations in CEA/CA 19-9 expression profiles within the reference range impact CRC recurrence.

## 1. Introduction

Colorectal cancer (CRC) is the third-most prevailing malignancy and the second-most prevailing cause of mortality, and its incidence continues to increase [1, 2]. The Global Cancer Statistics 2020 of the WHO Cancer Research Center reported that novel CRC cases in 2020 approached 1,880,000, with a mortality incidence rate approximating 920,000 [3]. Owing to increased early detection with cancer screening programs and advances in systemic treatment such as curative surgery, chemotherapy, vascular endothelial growth factor (VEGF)-targeted treatment (e.g., bevacizumab, cetuximab), and BRAF V600E/K-mutant targeted therapy, more patients survive after CRC treatment [4, 5].

Present monitoring recommendations for follow-up after CRC diagnosis include routine RAS/BRAF(V600E) status, physical examinations, and further symptom-related imaging tests [6, 7]. However, these clinical trials were mainly conducted using imaging-based methods having low sensitivity (such as CT), physical assessments having assessor-dependent subjective variations in sensitivity (such as abdominal sonography, digital rectal examination), or analytical platforms having restricted specificity (e.g., bone scan), excluding the use of tumor markers [8, 9].

The article "Elevated CEA and CA 19-9 Levels within the Normal Ranges Increase the Likelihood of CRC Recurrence in the Chinese Han Population" was retracted in 2023. Reasons: signs of a paper mill; suspected computer-generated content; unreliable results or conclusions; lack of ethics approval or compliance.

CEA/CA 19-9 are serum tumor biomarkers in CRC that are extensively deployed within clinic-based settings. CEA/CA 19-9 are non-invasive and easily available cancer biomarkers concerning CRC immediate monitoring/prediction during early, advanced, and metastatic CRC [10–12]. Notwithstanding, to the best of our knowledge, clinical values within the normal range have not been assessed. We hypothesized that changes in CEA/CA 19-9 expression profiles inside reference ranges could affect the recurrence of CRC; thus, the association between elevated CEA/CA 19-9 expression profiles inside reference ranges and CRC recurrence was analyzed within this investigation.

## 2. Materials and Methods

### 2.1. Ethical Approval

The Institutional Review Board of Hangzhou Ninth People's Hospital approved this study (IRB No. 2021-12-076) in line with the Declaration of Helsinki (2013) and did not request informed consent since solely anonymous data sets were regularly recorded during medical assessments.

### 2.2. CRC Patient Medical Profiles

This study enrolled CRC patients who had curative surgery followed by adjuvant treatment at Hangzhou Ninth People Hospital between January 2010 and January 2017. Because the objective consisted of evaluating prospective links across changes in CEA/CA 19-9 expression profiles and recurrence within cases having CEA/CA 19-9 inside the reference range at diagnosis, analyses focused solely on cases undergoing CEA/CA 19-9 expression profile examination on diagnoses (*n* = 3,265). Participants who had *CEA* > 5 ng/mL or *CA*19 − 9 > 40 U/mL at diagnosis (*n* = 493) and those who did not have a follow-up CEA or CA 19-9 (*n* = 176) were excluded. The final sample size was 2,596 (Figure 1).

#### 2.2.1. CEA/CA 19-9 Assays

An i2000 immunoassay analyzer (Abbott, Illinois, USA) was used to assess the serum CEA/CA, 19-9 levels, and chemiluminescence immunoassay (CLIA) was used to detect the outcomes. The reference ranges for CEA/CA 19-9 were 0–5 ng/mL and 0–40 U/mL, respectively.

### 2.3. Clinicopathological Features

Two experienced pathologists reviewed and determined the primary tumor characteristics. Retrospective analyses were subsequently performed in a non-stratified and non-matched manner. Clinicopathological features, including patient sex, age, pT/pN classification, histological subtype, location, tumor grade, vascular invasion, perineural invasion, metastases, and clinical stage of disease, were collected in line with Union for International Cancer Control (UICC). Recurrence was deemed an initial-detected event of local and/or distant CRC recurrence.

### 2.4. Statistical Analysis

GraphPad Prism 7™ (GraphPad Inc.TM, USA) was used for statistical analysis, and *P* < 0.05 was considered significant. Participants were enrolled on the day of surgery (baseline) and were followed up until the trial ended, death occurred, or the last available visit. The development of recurrence was the endpoint of the study. Patients were considered censored in the sensitivity analysis if they had CEA >5 ng/mL or CA19-9 >40 U/mL during the follow-up.

The article "Elevated CEA and CA 19-9 Levels within the Normal Ranges Increase the Likelihood of CRC Recurrence in the Chinese Han Population" was retracted in 2023. Reasons: signs of a paper mill; suspected computer-generated content; unreliable results or conclusions; lack of ethics approval or compliance.

Compared with previous examinations, study exposure changed within CEA/CA 19-9 expression profiles and was considered a time-varying variable. Using this time-dependent exposure design, the same person can contribute person-time to all change-level categories in each examination. The level of change per inspection contributed to the number of visits from the inspection date to the next inspection or final assessment. Hazard ratios (HRs) with 95% confidence intervals (CIs) were calculated for recurrence. To account for other potential confounders, we adjusted for sex, age, pT/pN classification, histological subtype, location, tumor grade, vascular invasion, perineural invasion, presence of metastases, and targeted therapy. Compared with previous examinations, changes within CEA/CA19-9 expression profiles were modeled as continuous variables for providing versatile estimates for dose–response association across shifts within CEA/CA19-9 expression profiles and recurrence.

## 3. Results

### 3.1. Patient Profiles

Mean (standard deviation, SD) age of investigation participants (*n* = 2596) was 61.4°years (8.6°years). The proportion of participants with ≥1 SD elevation within CEA or CA19-9 expression profiles throughout follow-up compared with the previous examination was 24.2% (*n* = 629) and 22.2% (*n* = 577), respectively. Compared with cases having raised *CEA* ≥ 1 SD or *CA*19 − 9 ≥ 1 SD, cases having stable CEA or CA19-9 expression profiles (change <1 SD) were less likely to have mucinous lesion (CEA: 28.9% *vs.* 2.8%, *P* < 0.001; CA19-9: 27.6% *vs.* 3.9%, *P* < 0.001), T3–T4 stage (CEA: 85.2% *vs.* 22.3%, *P* < 0.001; CA19-9: 77.6% *vs.* 26.1%, *P* < 0.001), lymph node metastasis (CEA: 93.3% *vs.* 71.0%, *P* < 0.001; CA19-9: 85.1% *vs.* 73.9%, *P* < 0.001), vascular invasion (CEA: 87.9% *vs.* 2.3%, *P* < 0.001; CA19-9: 81.6% *vs.* 6.3%, *P* < 0.001), less likely to receive treatment (chemotherapy: CEA: 83.1% *vs.* 69.8%, *P* < 0.001; CA19-9: 77.6% *vs.* 71.7%, *P* = 0.005; radiation therapy: CEA: 90.9% *vs.* 81.7%, *P* < 0.001; CA19-9: 94.3% *vs.* 81.0%, *P* < 0.001), and reduced expression profiles of CEA or CA19-9 at surgery (CEA: 2.6 ng/mL *vs.* 2.1 ng/mL, *P* < 0.001; CA19-9: 19.2 U/mL *vs.* 13.7 U/mL, *P* < 0.001).

### 3.2. HR for Recurrence Based on Changes in CEA/CA 19-9

During medical assessments (median follow-up =°5.2°years), 837 patients experienced recurrence. The incidence rates/100 person-years in participants having stable/elevated CEA expression profiles were 3.14 and 10.71, respectively. In comparison to cases having stable CEA expression profiles, cases having elevated CEA expression profiles (≥1 SD) were at higher risk for recurrence (HR = 7.06, 95%CI = 5.23–8.10; Table 1). The incidence rates per 100 person-years in participants with stable and elevated CA19-9 expression profiles were 2.93 and 7.62, respectively. Compared with patients with stable CA19-9 expression profiles, cases of elevated CA19-9 expression profiles (≥1 SD) were at higher risk for recurrence (HR = 3.98, 95%CI = 3.13–4.82; Table 2).

The article "Elevated CEA and CA 19-9 Levels within the Normal Ranges Increase the Likelihood of CRC Recurrence in the Chinese Han Population" was retracted in 2023. Reasons: signs of a paper mill; suspected computer-generated content; unreliable results or conclusions; lack of ethics approval or compliance.

### 3.3. Subgroup Analysis for HR for Recurrence Based on Changes in CEA/CA 19-9

Subtype analyses demonstrated raised CEA/CA 19-9 to be linked to mucinous subtype, T stage, lymph node metastases, and vascular invasion (Table 3). Furthermore, the association was stronger for cases with T3–T4 stage and cases with mucinous subtype, lymph node metastases, and vascular invasion than for cases with T1–T2 stage and cases without mucinous subtype, lymph node metastasis, and vascular invasion (*P*-value for interaction <0.05). In spline regression models, the associations between changes in CEA/CA 19-9 expression profiles and recurrence incidences were nonlinear, with stronger associations when CEA/CA 19-9 expression profiles were raised in comparison to decreased expression profiles (*P*-value for nonlinear spline terms <0.05; Figure 2).

## 4. Discussion

This investigation analyzed changes in CEA/CA 19-9 expression profiles within 2,596 CRC patients, with significant associations found between elevated CEA/CA 19-9 expression profiles inside the reference range and recurrence. Associations between raised CEA/CA 19-9 expression profiles and recurrence were observed across all pathological tumor stages and progression.

In numerous studies, elevated CEA/CA 19-9 expression profiles have been linked to CRC prognosis in various ranges and situations. In metastatic CRC cases, elevated CEA/CA 19-9 expression profiles showed poor overall survival [13, 14]. CRC cases having bone metastasis, which shows a better prognosis among metastatic CRC cases, also had elevated CEA/CA 19-9 expression profiles and significantly poor progression-free survival [15, 16]. Furthermore, in many studies, stage I–III CRC cases having elevated CEA/CA 19-9 expression profiles had poor disease-free survival [17–20]. In previous studies, fewer than 1,000 patients were reported, and cases with CEA or CA 19-9 beneath the cutoff value were ignored. This investigation included many operable cases with CEA or CA 19-9 below the cutoff value (mean CEA: 5 ng/mL; mean CA 19-9: 40.0 U/mL), and changes below the cutoff value were analyzed.

The article "Elevated CEA and CA 19-9 Levels within the Normal Ranges Increase the Likelihood of CRC Recurrence in the Chinese Han Population" was retracted in 2023. Reasons: signs of a paper mill; suspected computer-generated content; unreliable results or conclusions; lack of ethics approval or compliance.

Although current guidelines do not recommend routine imaging such as abdominal CT or bone scans to detect distant metastasis in asymptomatic CRC patients, many clinicians routinely use intensive imaging and tumor biomarkers (CA 19-9, CEA, CA-242) to detect distant metastasis [10, 13, 14]. Because clinical trials conducted decades ago demonstrated scarce benefits for routine intensive imaging and do not reflect recent modern imaging and target therapies, routine intensive imaging is currently used to detect distant metastases [21]. Furthermore, the survival of cases with metastatic CRC has markedly ameliorated throughout the preceding few decades, and some cases with metastatic CRC, especially oligometastases, enjoy prolonged clinical remission if given intensive treatment [22]. Similarly, the European Society for Medical Oncology (ESMO) and the American Society of Clinical Oncology (ASCO) do not advise serial measurements for CEA/CA 19-9 during the medical assessment of early CRC due to the lack of data indicating that it increases survival benefit [23]. However, compared to CT or bone scans, which can potentially harm patients, CEA/CA 19-9 remain very non-invasive, easily available, and cost-effective tumor biomarkers. Many clinicians use a serial assessment of tumor biomarkers, including CEA/CA 19-9, as part of routine medical assessments in asymptomatic, early CRC cases.

In the current study, elevated CEA or CA 19-9 expression profiles with inside reference range were associated with worse disease-free survival. Recently, liquid biopsy based on circulating tumor DNA (ctDNA) or cell-free DNA is an emerging new technique for diagnosing and monitoring CRC [24, 25]. Because data on CEA/CA 19-9 are sufficient, a future investigation comparing ctDNA with CEA/CA 19-9 is warranted.

This investigation has several limitations. First, this was a retrospective investigation conducted at a single institution, which limits the generalizability of the results. Second, other tumor biomarkers such as CA242 were not analyzed; thus, the risk of recurrence could not be compared with other tumor biomarkers. External validation and comparison with other tumor biomarkers are necessary. Third, the associations across CEA or CA 19-9 level and a detailed recurrence pattern, such as distant metastasis and locoregional recurrence, were not demonstrated. Similarly, the correlation between CEA or CA 19-9 level and overall survival was not observed, and further studies are necessary. However, we used a time-dependent exposure design in which the same individual can contribute person-time to all change-level categories in each examination, which was conducted with a large homogenous CRC patient cohort, and the first in which elevated CEA or CA 19-9 level with inside reference range were shown to affect CRC recurrence.

The article "Elevated CEA and CA 19-9 Levels within the Normal Ranges Increase the Likelihood of CRC Recurrence in the Chinese Han Population" was retracted in 2023. Reasons: signs of a paper mill; suspected computer-generated content; unreliable results or conclusions; lack of ethics approval or compliance.

## 5. Conclusion

In conclusion, changes in CEA/CA 19-9 expression profiles with inside reference range affect CRC recurrence. Whether early detection of changes in CEA/CA 19-9 expression profiles with inside reference range can improve disease-free survival should be investigated in future studies.

## Figures and Tables

**Figure 1:** Schematic diagram for patient inclusion.

**Figure 2:** Recurrence hazard ratio (HR) adjusted for variations in CEA/CA 19-9 expression profiles. (a) HR adjusted for variations in CEA level. (b) HR adjusted for CA 19-9 level changes.

**Table 1:** Characteristics of study participants.

Characteristics	Overall	CEA (ng/mL)				CA19-9 (U/mL)			
		Stable	1 SD elevated^a^	*t*/*χ*^2^	*P*	Stable	1 SD elevated^a^	*t*/*χ*^2^	*P*
***n***	2596	1967	629			2019	577		
**Baseline levels (mean, SD)**	**CEA:** 2.2 (0.8) ng/mL; **CA19-9:** 14.9 (7.3) U/mL	2.1 (0.6)	2.6 (0.9)	–15.940	<0.001	13.7 (6.7)	19.2 (7.5)	–16.921	<0.001
**Age, years (mean, SD)**	61.4 (8.6)	61.4 (8.7)	61.2 (8.4)	0.506	0.613	61.4 (8.8)	61.3 (8.5)	0.052	0.959
**Sex**				0.188	0.664			0.038	0.845
Female (%)	873	657 (33.4)	216 (34.3)			677 (33.5)	196 (34.0)		
Male (%)	1723	1310 (66.6)	413 (65.7)			1342 (66.5)	381 (66.0)		
**The anatomic site of the tumor**				7.436	0.024			1.994	0.369
Right-sided (%)	762	574 (29.2)	188 (29.9)			606 (30.0)	156 (27.0)		
Left-sided (%)	336	236 (12.0)	100 (15.9)			257 (12.7)	79 (13.7)		
Rectal cancers	1498	1157 (58.8)	341 (54.2)			1156 (57.3)	342 (59.3)		
**Mucinous subtype**				392.510	<0.001			303.656	<0.001
No (%)	2359	1912 (97.2)	447 (71.1)			1941 (96.1)	418 (72.4)		
Yes (%)	237	55 (2.8)	182 (28.9)			78 (3.9)	159 (27.6)		
**T stage**				805.569	<0.001			509.502	<0.001
T1–T2 (%)	1622	1529 (77.7)	93 (14.8)			1493 (73.9)	129 (22.4)		
T3–T4 (%)	974	438 (22.3)	536 (85.2)			526 (26.1)	448 (77.6)		
**Lymph node metastasis**				131.556	<0.001			30.953	<0.001
No (%)	612	570 (29.0)	42 (6.7)			526 (26.1)	86 (14.9)		
Yes (%)	1984	1397 (71.0)	587 (93.3)			1493 (73.9)	491 (85.1)		
**Vascular invasion**				1966.467	<0.001			1433.108	<0.001
No (%)	1997	1921 (97.7)	76 (12.1)			1891 (93.7)	106 (18.4)		
Yes (%)	599	46 (2.3)	553 (87.9)			128 (6.3)	471 (81.6)		
**Chemotherapy**				43.106	<0.001			7.998	0.005
No (%)	700	594 (30.2)	106 (16.9)			571 (28.3)	129 (22.4)		
Yes (%)	1896	1373 (69.8)	523 (83.1)			1448 (71.7)	448 (77.6)		
**Radiation therapy**				29.906	<0.001			58.551	<0.001
No (%)	416	359 (18.3)	57 (9.1)			383 (19.0)	33 (5.7)		
Yes (%)	2180	1608 (81.7)	572 (90.9)			1636 (81.0)	544 (94.3)		

^a^Elevated ≥1 SD of baseline CEA (0.8) or CA 19-9 (7.3).

The article "Elevated CEA and CA 19-9 Levels within the Normal Ranges Increase the Likelihood of CRC Recurrence in the Chinese Han Population" was retracted in 2023. Reasons: signs of a paper mill; suspected computer-generated content; unreliable results or conclusions; lack of ethics approval or compliance.

**Table 2:** HR for recurrence based on changes in CEA and CA 19-9.

Tumor markers	Change between previous examination and current examination	Number of recurrences (incidence rate per 100 person-years)	Unadjusted HR (95% CI)	Adjusted HR (95% CI)^b^
**CEA**				
	Stable	434 (3.14)	Reference	Reference
	Elevated ≥1 SD ^a^	403 (10.71)	7.95 (5.49–10.99)	7.06 (5.23–8.10)
**CA19-9**				
	Stable	472 (2.93)	Reference	Reference
	Elevated ≥1 SD ^a^	365 (7.62)	4.72 (3.34–6.23)	3.98 (3.13–4.82)

^a^Adjusted for sex, age, pT/pN classification, histological subtype, location, tumor grade, vascular invasion, perineural invasion, presence of metastases, and targeted therapy.

^b^Elevated ≥1 SD of baseline CEA (0.8) or CA 19-9 (7.3).

**Table 3:** Subgroup analysis for HR for recurrence based on changes in CEA and CA 19-9.

Change between previous examination and current examination	Elevated ≥1 SD CEA		Elevated ≥1 SD CA19-9	
	Unadjusted HR (95% CI)	Adjusted HR (95% CI)^a^	Unadjusted HR (95% CI)	Adjusted HR (95% CI)^a^
**Gender**				
Female (%)	1.03 (0.89–1.16)	0.98 (0.93–1.02)	1.01 (0.98–1.03)	1.00 (0.98–1.03)
Male (%)	1.01 (0.94–1.08)	1.02 (0.97–1.06)	1.03 (0.97–1.07)	0.98 (0.95–1.01)
*P-*Value for interaction	0.904	0.847	0.923	0.951
**The anatomic site of the tumor**				
Right-sided (%)	0.97 (0.94–1.01)	0.99 (0.96–1.03)	1.01 (0.96–1.07)	0.97 (0.93–1.01)
Left-sided (%)	1.07 (1.02–1.13)	1.01 (0.97–1.05)	1.03 (0.99–1.06)	1.00 (0.98–1.03)
Rectal cancers	0.99 (0.97–1.01)	1.00 (0.98–1.03)	0.98 (0.96–1.01)	1.01 (0.99–1.04)
*P*-Value for interaction	0.644	0.897	0.830	0.795
**Mucinous subtype**				
No (%)	1.43 (1.17–1.76)	1.95 (1.05–3.04)	2.07 (1.69–2.53)	1.58 (1.06–2.38)
Yes (%)	2.12 (1.73–2.64)	8.82 (6.73–10.31)	2.53 (1.95–3.84)	4.87 (2.47–7.70)
*P*-Value for interaction	0.017	<0.001	0.025	<0.001
**T stage**				
T1–T2 (%)	1.19 (1.14–1.32)	1.38 (1.09–2.57)	1.07 (1.02–1.15)	1.45 (1.37–1.82)
T3–T4 (%)	3.15 (2.47–4.10)	5.82 (3.16–8.13)	1.61 (1.21–2.09)	3.78 (2.42–5.17)
*P*-Value for interaction	0.001	<0.001	0.037	0.003
**Lymph node metastasis**				
No (%)	1.34 (1.09–1.74)	2.73 (2.11–4.05)	1.21 (1.04–1.39)	2.07 (1.59–2.90)
Yes (%)	4.02 (3.66–4.96)	8.64 (4.06–13.56)	2.97 (2.23–4.11)	6.12 (4.09–9.13)
*P-*Value for interaction	<0.001	<0.001	0.009	<0.001
**Vascular invasion**				
No (%)	1.76 (1.38–2.37)	2.41 (1.61–3.39)	1.44 (1.13–1.89)	1.84 (1.27–2.65)
Yes (%)	4.04 (2.50–6.84)	6.00 (4.21–8.57)	2.88 (1.89–4.05)	2.96 (1.75–4.37)
*P*-Value for interaction	0.005	<0.001	0.012	0.003

^a^Adjusted for sex, age, pT/pN classification, histological subtype, location, tumor grade, vascular invasion, perineural invasion, presence of metastases, and targeted therapy.

The article "Elevated CEA and CA 19-9 Levels within the Normal Ranges Increase the Likelihood of CRC Recurrence in the Chinese Han Population" was retracted in 2023. Reasons: signs of a paper mill; suspected computer-generated content; unreliable results or conclusions; lack of ethics approval or compliance.

## Data Availability

The data used to support the findings of this study are available from the authors upon request.
